# Comprehensive Analysis of LncRNA AC010789.1 Delays Androgenic Alopecia Progression by Targeting MicroRNA-21 and the Wnt/*β*-Catenin Signaling Pathway in Hair Follicle Stem Cells

**DOI:** 10.3389/fgene.2022.782750

**Published:** 2022-02-15

**Authors:** Jiachao Xiong, Baojin Wu, Qiang Hou, Xin Huang, Lingling Jia, Yufei Li, Hua Jiang

**Affiliations:** ^1^ Department of Plastic Surgery, Shanghai East Hospital, Tongji University School of Medicine, Shanghai, China; ^2^ Department of Plastic Surgery, Huashan Hospital, Fudan University, Shanghai, China; ^3^ Department of Dermatology, Tongji Hospital, Tongji University School of Medicine, Shanghai, China

**Keywords:** androgen alopecia, hair follicle stem cells, AC010789.1, Wnt/β-catenin, TGF-1

## Abstract

**Background:** Androgen alopecia (AGA), the most common type of alopecia worldwide, has become an important medical and social issue. Accumulating evidence indicates that long noncoding RNAs (lncRNAs) play crucial roles in the progression of various human diseases, including AGA. However, the potential roles of lncRNAs in hair follicle stem cells (HFSCs) and their subsequent relevance for AGA have not been fully elucidated. The current study aimed to explore the function and molecular mechanism of the lncRNA AC010789.1 in AGA progression.

**Methods:** We investigated the expression levels of AC010789.1 in AGA scalp tissues compared with that in normal tissues and explored the underlying mechanisms using bioinformatics. HFSCs were then isolated from hair follicles of patients with AGA, and an AC010789.1-overexpressing HFSC line was produced and verified. Quantitative real-time polymerase chain reaction (qRT-PCR) and Western blotting were performed to verify the molecular mechanisms involved.

**Results:** AC010789.1 overexpression promoted the proliferation and differentiation of HFSCs. Mechanistically, we demonstrated that AC010789.1 overexpression promotes the biological function of HFSCs by downregulating miR-21-5p and TGF-*β*1 expression but upregulating the Wnt/*β*-catenin signaling pathway.

**Conclusion:** These results reveal that overexpression of AC010789.1 suppresses AGA progression via downregulation of hsa-miR-21-5p and TGF-*β*1 and promotion of the Wnt/*β*-catenin signaling pathway, highlighting a potentially promising strategy for AGA treatment.

## Introduction

Alopecia, a common disorder occurring worldwide, characterized by hair loss, can be caused by multiple factors, such as heredity, hormonal disorders, immune inflammation, malnutrition, environmental factors, mental disorders, and aging (Ho and Shapiro, 2019). Androgen alopecia (AGA) is the most common type of alopecia and has become an important medical and social issue due to its high incidence; increasingly young onset age; and associated psychological problems, such as depression, anxiety, and emotional disorders (Bas et al., 2015; Molina-Leyva et al., 2016; Katzer et al., 2019; Ding et al., 2020). Currently, finasteride and minoxidil are the only therapeutic drugs approved by the Food and Drug Administration for AGA treatment (Chen et al., 2020a). Finasteride, a specific inhibitor of type II 5*α* reductase, inhibits the metabolic conversion of testosterone to highly active dihydrotestosterone, reducing the effect of active androgens on hair follicles (Spinucci and Pasquali, 1996). However, finasteride is associated with a risk of sexual dysfunction and depression during treatment (Motofei et al., 2020). Minoxidil treats AGA by predominantly promoting hair growth but can cause side effects, such as contact dermatitis, skin irritation, and dizziness during treatment, and on treatment cessation, alopecia generally recurs (Goren et al., 2017; Jimenez-Cauhe et al., 2019). Hair transplantation is the gold standard for AGA treatment, but the limited number of active hair follicles in the donor site makes it impossible to apply to large areas of baldness (Chouhan et al., 2019a; Chouhan et al., 2019b). Hence, new methods for the treatment of AGA need to be developed urgently.

The three phases of periodic hair follicle growth are resting, growth, and degenerative periods, and cessation of this regeneration cycle is the main mechanism contributing to AGA (Baker and Murray, 2012). Previous studies report that the periodic growth of hair follicles depends on the hair follicle stem cells (HFSCs) located in the bulge area of the hair follicle (Cotsarelis et al., 1990; Fu and Hsu, 2013). HFSCs are a group of adult stem cells with self-renewal ability that specifically express surface markers such as CD34 and CK15 (Morris et al., 2004; Owczarczyk-Saczonek et al., 2018). In normal conditions or during wound repair, HFSCs in the bulge area activate and differentiate into various hair follicle cell types for hair follicle regeneration (Oshima et al., 2001; Yang et al., 2017). However, there is evidence that the scalp hair follicles in patients with AGA are impaired in HFSC activation, thereby preventing their differentiation into hair follicle precursors. Garza et al. (2011) found that, although patients with AGA had a similar quantity of hair follicles in the alopecia scalp area as in nonalopecia areas, the HFSCs in the alopecia areas were in a static state and did not actively differentiate into hair follicle precursors. Thus, activation of HFSC proliferation and differentiation may be an effective breakthrough for the treatment of AGA.

Long noncoding RNAs (lncRNAs), a type of noncoding RNA over 200 nt in length, have attracted considerable interest in recent years. Functional data suggest that they play essential regulatory roles in multiple biological processes, such as cell development, differentiation, disease, subcellular localization, and cell structure maintenance (Yao et al., 2019). Intriguingly, genome analyses comparing AGA scalp tissues with adjacent normal tissues (defined as 5 cm from the margin of the AGA areas with a follicle density >325/cm^2^) in patients with AGA found a large number of differentially expressed lncRNAs, indicating that the dysregulation of lncRNA expression profiles may be involved in AGA progression (Chew et al., 2016; Bao et al., 2017). Moreover, several lines of evidence demonstrate a novel lncRNA regulatory mechanism in promoting hair follicle regeneration. Zhu et al. (2020) demonstrate that overexpression of lncRNA H19 can directly downregulate the expression of Wnt pathway inhibitors, including DKK1, Kremen2, and sFRP2, which activates Wnt signaling, thereby maintaining the hair follicle regeneration potential of dermal papilla cells (DPCs). Likewise, Lin et al. (2020a); Lin et al. (2020b) found that lncRNA XIST targets miR-424 and PCAT1 targets miR-329 to activate Wnt and hedgehog signaling, respectively, and maintain the regeneration characteristics of DPCs. To date, many molecular mechanisms of DPC-mediated hair follicle regeneration have been investigated. However, the role of the potential connection between lncRNAs and HFSCs in AGA has not been fully elucidated.

The current study aimed to explore the potential function of the lncRNA AC010789.1 in AGA progression. We demonstrate that AC010789.1 expression was downregulated in AGA scalp tissues, and overexpression of AC010789.1 promoted the proliferation and differentiation of HFSCs. Mechanistically, overexpression of AC010789.1 was shown to delay AGA progression by interacting with miR-21 and activating Wnt/*β*-catenin signaling. Therefore, this study provides insights into the mechanisms underlying AC010789.1 regulation of AGA progression to provide a new theoretical and experimental basis for the prevention and treatment of AGA.

## Materials and Methods

### Tissue Collection and Ethics Statement

Hair follicle tissues extracted from patients with AGA were obtained from the Shanghai East Hospital affiliated with the Tongji University School of Medicine, and informed consent was obtained from all patients. Ethical approval was obtained from the Shanghai East Hospital Ethics Committee. Tissue specimens were snap-frozen and stored in liquid nitrogen until further use.

### Microarray Data Acquisition

Gene expression microarray data sets (GSE84839 and GSE36169) were downloaded from the Gene Expression Omnibus (GEO) database (https://www.ncbi.nlm.nih.gov/geo). The GSE84839 data set was based on the GPL21827 platform (Agilent-079487 Arraystar Human LncRNA microarray V4) and included three pairs of male AGA scalp tissues and adjacent normal tissues. The GSE36169 data set was based on the GPL96 platform (Affymetrix Human Genome U133A Array) and contained AGA and adjacent normal scalp tissues from five individuals. The lncRNA and mRNA expression data in the AGA and adjacent normal tissues were downloaded and used for this study.

### Differential Analysis of lncRNA and mRNA Expression

Differential analysis of lncRNA and mRNA expression between AGA and adjacent normal scalp tissues was performed using the GEO2R analysis tool. The platform data were converted using R language software and standardized using the limma array function within the R package (http://www.bioconductor.org/). A *p*-value < .05, and a base-2 logarithm of fold change (log FC) < −1 or >1 were used as selection criteria to screen differentially expressed lncRNAs and mRNAs (Xiong et al., 2020).

### Functional and Pathway Enrichment Analysis

Database for Annotation, Visualization, and Integrated Discovery (DAVID) v6.8 (https://david.ncifcrf.gov/) provides a comprehensive annotation tool to help investigators better clarify the biological function of the submitted genes (Dennis et al., 2003). In this study, DAVID v6.8 was used for gene ontology (GO) annotation and Kyoto Encyclopedia of Genes and Genomes (KEGG) pathway enrichment analysis. GO annotation analysis revealed biological processes (BPs), cellular components (CCs), and molecular functions (MFs) of the genes. Statistical significance was set at *p* < 0.05. Then, XTalkDB (http://www.xtalkdb.org/home), a database that documents scientific literature supporting crosstalk between pairs of signaling pathways, was used to explore the relationship between pathways.

### Integrated Analysis of Interaction Network

GeneMANIA (http://genemania.org/) is a data set that provides a series of functional association information to identify the relation between genes of the submitted set in terms of their genetic interactions, pathways, expression patterns, localization, and protein domain similarity. In this study, protein-protein interaction (PPI) networks were analyzed using the GeneMANIA data set, and Cytoscape (version 3.7.2) was used to visualize the PPI networks.

### Isolation and Cultivation of HFSC

Isolation of HFSCs was performed as previously described (Aran et al., 2020). Follicular unit extraction was performed to collect and isolate hair follicle tissues from 20 patients with AGA under a stereomicroscope. A needle was used to separate the hair shaft and papilla, and only the bulge areas were reserved. The bulge areas were treated with dispase II (2.5 mg/ml, Sigma, United States) and collagenase I (1 mg/ml, Gibco, United States) for 60 min, and 0.25% trypsin-ethylene diamine tetra acetic acid (EDTA; Gibco, Grand Island, NY, United States) for 15 min. The obtained cells were cultured in a keratinocyte serum-free medium (K-SFM, Gibco) in a 5% CO_2_ humidified incubator at 37°C, and the medium was changed every 2–3 days. The third passage (P3) of HFSCs was characterized by immunofluorescence with an anti-K15 antibody (Santa Cruz Biotechnology, TX, United States) and was used for follow-up studies.

### Cell Proliferation Assay

Cell Counting Kit 8 (CCK8) assays (Beyotime Biotechnology Company, Jiangsu, China) and 5-ethynyl-2 deoxyuridine (EdU) assays (RiboBio, Guangzhou, China) were performed to assess the cell proliferation ability. For CCK8 assays, cells were seeded at approximately 2×10^3^ cells/well in 96-well plates, and cell attachment was allowed for 12 h. Then, a 10 μl CCK8 test solution was added to each well at 24, 48, 72, and 96 h, and the cells were incubated in a humidified incubator with 5% CO_2_ at 37°C for 2 h at each time point to evaluate the cell growth viability. The optical density (OD) was measured at 450 nm with a microplate reader (Tecan, Thermo Scientific, United States). For EdU assays, the experiments were performed according to the manufacturer’s instructions (Xiong et al., 2019). Then, the cells were observed under a fluorescence microscope (Zeiss HLA100, Shanghai, China) and analyzed by using ImageJ software (Bethesda, MD, United States). The data shown are representative of three independent experiments.

### Quantitative Real-Time Polymerase Chain Reaction

Total RNA was isolated from tissues or cells using Trizol^®^ Reagent (Life Technologies, United States) and reverse transcribed into cDNA using a cDNA synthesis kit (Thermo Scientific) according to the manufacturer’s instructions. qRT-PCR was performed as previously reported (Xiong et al., 2019). Melt curves were established for the reactions, and the normalized fold expression was calculated using the 2^−ΔΔ Ct^ method. The primer sequences are listed in Table 1.

**TABLE 1:** Primers used for qRT-PCR.

Gene	Forward primer (5′-3′)	Reverse primer (5′-3′)
GAPDH	AGAAGGCTGGGGCTCATT	TGC​TAA​GCA​GTT​GGT​GGT​G
AC010789.1	TGC​ATC​CCT​GGC​AAT​ACT​CAG	GGA​GTG​CTG​TGC​ATT​CAT​TGG
U6	CGA​TAC​AGA​GAA​GAT​TAG​CAT​GGC	AAC​GCT​TCA​CGA​ATT​TGC​GT
hsa-miR-21-5p	GCA​GTA​GCT​TAT​CAG​ACT​GAT​G	AGT​GCG​TGT​CGT​GGA​GTC​G
TGF-*β*1	ATG​GAG​AGA​GGA​CTG​CGG​AT	GTA​GTG​TTC​CCC​ACT​GGT​CC
K6hf	TTG​TAG​CCC​TGA​AAA​AGG​ACG	CAG​CTC​TGC​ATC​AAA​GAC​TGA​G
WNT10b	CAT​CCA​GGC​ACG​AAT​GCG​A	CGG​TTG​TGG​GTA​TCA​ATG​AAG​A
DKK-1	GAG​TAC​TGC​GCT​AGT​CCC​AC	TTT​GCA​GTA​ATT​CCC​GGG​GC

### Western Blotting

The cells from each sample were collected and lysed in radioimmunoprecipitation (RIPA) buffer (Thermo Scientific), followed by centrifugation at 1,200×*g* for 10 min and subsequent collection of the supernatant. Western blotting was performed as previously described (Xiong et al., 2019). The primary antibodies were GAPDH (1:20,000, Proteintech, China), Lgr5 (1:1,000, Abcam, United States), TGF-*β*1 (1:1,000, Santa Cruz Biotechnology, United States), and *β*-catenin (1:1,000, Cell Signaling Technology, United States), and the secondary antibody was horseradish peroxidase-conjugated goat antimouse (1:10,000, Abcam, United States). Protein expression was observed and visualized by chemiluminescence using an Alpha Imager scanner (Tecan, Thermo Scientific).

### Statistical Analysis

All data are expressed as the mean ± standard deviation, and statistical significance was determined using Student’s *t*-test. All statistical analyses were performed using SPSS (version 17.0). Statistical significance was set at *p* < 0.05.

## Results

### AC010789.1 Expression is Downregulated in Patients With AGA

To investigate the role of lncRNAs in AGA, we used the gene expression microarray data set GSE84839, which included the data of three pairs of male scalp AGA and adjacent normal tissues. Analysis using the screening criteria of *p* < 0.05 and |log FC| > 1 revealed a total of 4,939 differentially expressed lncRNAs (4,239 upregulated and 700 downregulated). A volcano map was used to show the distribution of all differentially expressed lncRNAs (Figure 1A). AC010789.1, whose expression was significantly reduced in AGA scalp tissues compared with adjacent normal tissues, was selected for further analysis. To validate the results from the GSE84839 data set, we examined the expression level of AC010789.1 in clinical AGA scalp and adjacent normal tissues. The results showed that AC010789.1 expression was indeed downregulated in the AGA scalp tissues of patients (Figure 1B). These results strongly indicate that AC010789.1 expression is significantly downregulated in AGA scalp tissues and might be an essential predictive factor for patients with AGA.

**FIGURE 1:** AC010789.1 is downregulated in patients with AGA, and its overexpression promotes proliferation and differentiation of HFSCs. **(A)** Volcano plot of the GSE84839 microarray data set. **(B)** AC010789.1 was downregulated in scalp tissues compared with adjacent normal tissues of AGA patients. *n* = 6 **(C)** The HFSCs highly express K15. HFSCs were stained with green fluorescence, and all nuclei were stained with blue fluorescence. Scale bars indicate 100 μm. **(D)** The AC010789.1 overexpression HFSC cell lines were successfully constructed. **(E–I)** Overexpression of AC010789.1 increased cell abilities of differentiation and proliferation. Scale bars indicate 100 μm *n* = 3 *p < 0.05, **p < 0.01 and ***p < 0.001.

### Overexpression of AC010789.1 Promotes Proliferation and Differentiation of HFSCs

HFSCs were isolated from normal hair follicle tissues, and immunofluorescence was performed to detect the hair follicle stem cell marker K15. As shown in Figure 1C, the HFSCs displayed a high expression of K15. To better understand the biological effects of AC010789.1 on AGA development, we constructed an AC010789.1 overexpression plasmid, which was subsequently transfected into HFSCs. The qRT-PCR results in Figure 1D show that AC010789.1 was successfully overexpressed, and the resulting HFSC line (AC010789.1-OE) was used for further study. The qRT-PCR analysis showed that overexpression of AC010789.1 significantly upregulated the expression of HFSC differentiation markers K6HF and Lgr5 (Figures 1E,F). Subsequently, CCK8 and EdU assays revealed that AC010789.1 upregulation also resulted in increased cell proliferation (Figures 1G–I). Taken together, these experiments reveal that AC010789.1 has important functions in regulating the proliferation and differentiation of HFSCs.

### AC010789.1 Interacts With miR-21 to Participate in AGA Progression

LncRNAs can act as miRNA sponges to regulate downstream targets. Therefore, we predicted putative candidate AC010789.1-binding miRNAs using RNAhybrid v2.2 and identified hsa-miR-21-5p as a potential candidate (Figure 2A). Next, we demonstrated that the expression level of hsa-miR-21-5p negatively correlated with that of AC010789.1 in AC010789.1-OE samples (Figure 2B). Hence, we considered hsa-miR-21-5p to be a potential target of AC010789.1.

**FIGURE 2:** AC010789.1 interacts with miR-21 to participate in AGA progress and exploration on the pathogenesis of AGA. **(A)** RNAhybrid v2.2 showed the putative binding sites of miR-21-5p on AC010789.1. **(B)** Relative expression of miR-21-5p in AC010789.1-OE. *n* = 6 **(C)** Volcano plot of the GSE36169 microarray data set. **(D)** Venn diagram of upregulated and downregulated DEGs among the mRNA expression profiling sets GSE36169 and hsa-miR-21-5p targeted genes. *p < 0.05, **p < 0.01 and ***p < 0.001.

To further evaluate the mechanism by which AC010789.1 interacts with hsa-miR-21-5p in the pathogenesis of AGA, we analyzed the gene expression microarray data set GSE36169, which contained data of AGA and adjacent normal scalp tissues from five individuals. Analysis using the same screening criteria described above revealed a total of 198 differentially expressed genes (DEGs; 68 upregulated and 300 downregulated), which were represented on a volcano map (Figure 2C). Subsequently, we used the databases miRWalk and miRDB to predict the target genes of hsa-miR-21-5p and Venn diagram software to identify the genes that were common to both sets of analyses (Figure 2D). A total of 11 common genes (four upregulated and nine downregulated) were detected (Table 2).

**TABLE 2:** Common genes crossed by DEGs and hsa-miR-21-5p target genes.

Gene name	Regulated
ENPP4	Upregulated
JCHAIN	Upregulated
PLP1	Upregulated
P2RY14	Upregulated
LEF1	Downregulated
BNC2	Downregulated
SPOCK1	Downregulated
THBS1	Downregulated
TIMP3	Downregulated
VSNL1	Downregulated
FGF18	Downregulated

### GO Annotation and KEGG Pathway Enrichment Analysis of DEGs

To further explore the pathogenesis of AGA, we performed GO and KEGG enrichment analyses to further reveal the enrichment status of the DEGs in terms of their MFs, BPs, CCs, and pathways. With regard to BPs (Figures 3A,E), the upregulated DEGs were mainly involved in GO:0050776 (regulation of immune response), GO:0030199 (collagen fibril organization), and GO:0006954 (inflammatory response), and the downregulated DEGs were mainly involved in GO:0008544 (*epidermis* development), GO:0001942 (hair follicle development), and GO:0007010 (cytoskeleton organization). In terms of CCs (Figures 3B,F), the majority of upregulated DEGs were components of GO:0005576 (extracellular region), GO:0005615 (extracellular space), and GO:0072562 (blood microparticles), and the downregulated DEGs were mainly components of GO:0005882 (intermediate filament), GO:0045095 (keratin filament), and GO:0005615 (extracellular space). For the MFs (Figures 3C,G), the upregulated DEGs were mainly involved in GO:0031720 (haptoglobin binding), GO:0004252 (serine-type endopeptidase activity), and GO:0048407 (platelet-derived growth factor binding), and the downregulated DEGs were mainly involved in GO:0005198 (structural molecule activity), GO:0005509 (calcium ion binding), and GO:0008013 (beta-catenin binding). KEGG pathway analysis was used to explore pathway enrichment of the DEGs (Figures 3D,H). The most upregulated DEGs were significantly enriched in hsa05143 (African trypanosomiasis), hsa05144 (malaria), and hsa05150 (*Staphylococcus aureus* infection), and the downregulated DEGs were mainly enriched in hsa05144 (malaria), hsa04151 (PI3K-Akt signaling pathway), and hsa04350 (TGF-beta signaling pathway).

**FIGURE 3:** GO annotation and KEGG pathway enrichment analysis of the DEGs through the DAVID database. **(A,E)** The category of “biological process” of upregulated DEGs and downregulated DEGs, respectively. **(B,F)** The category of “cellular component” of upregulated DEGs and downregulated DEGs, respectively. **(C,G)** The category of “molecular function” of the predicted TG of upregulated DEGs and downregulated DEGs, respectively. **(D,H)** The category of “KEGG” of upregulated DEGs and downregulated DEGs, respectively.

### Comprehensive Analysis of the Common DEGs

Next, the PPI networks of the common DEGs were analyzed using GeneMANIA, and the 20 most relevant genes were identified. GPM6B, SOX10, MBP, PIM2, CDH19, PMP2, GPM6A, PTPRN, MAG, TNFRSF17, ENPP6, ENPP2, SP2, ITGAV, SPI1, PIGO, CD79A, ENPP7, PIGG, and ENPP5 were primarily associated with the PPI network of the upregulated common genes (Figure 4A), and COL6A1, GABRD, MLLT10, MFAP5, SGK1, RAI14, DDX17, HOXC4, MMP14, ADH1B, VAV2, EFNA5, PLA2G15, RAB31, PCK1, HOXA10, NRP1, ZKSCAN5, MBTPS2, and PRRX1 were primarily associated with the PPI network of the downregulated common genes (Figure 4B). Furthermore, all the common DEGs and their 20 most relevant network genes were analyzed by GO and KEGG enrichment analysis. For BP (Figure 4C), most of the genes were involved in GO:0002040 (sprouting angiogenesis), GO:0035987 (endodermal cell differentiation), and GO:0001525 (angiogenesis). For CC (Figure 4D), the genes were mainly components of GO:0005886 (plasma membrane) and GO:0031012 (extracellular matrix). With regard to MF (Figure 4E), a majority of the genes were involved in GO:0003705 (transcription factor activity, RNA polymerase II distal enhancer sequence-specific binding), GO:0019911 (structural constituent of myelin sheath), and GO:0002020 (protease binding). KEGG pathway enrichment analysis results showed that hsa04151 (PI3K-Akt signaling pathway) and hsa05221 (acute myeloid leukemia) were the most significantly enriched pathways of the genes (Figure 4F).

**FIGURE 4:** Comprehensive analysis of the common DEGs. **(A)** PPI network of the upregulated common DEGs. **(B)** PPI network of the downregulated common DEGs. **(C)** The category of “biological process” of the common DEGs and their most relevant genes. **(D)** The category of “cellular component” of the common DEGs and their most relevant genes. **(E)** The category of “molecular function” of the common DEGs and their most relevant genes. **(F)** The category of “KEGG” of the common DEGs and their most relevant genes.

### AC010789.1 Targets the Wnt/*β*-Catenin Signaling Pathway to Regulate AGA Progression

According to the results of KEGG pathway enrichment analysis, a majority of the enriched pathways were highly associated with Wnt/β-catenin signaling (Figures 5A,B). Thus, we analyzed the mRNA and protein expression levels of several key genes of the Wnt/β-catenin pathway, including DKK-1, TGF-*β*1, Wnt10b, and *β*-catenin in AC010789.1-OE. The results showed that the expression of DKK-1 and TGF-*β*1 was significantly downregulated, whereas the expression of Wnt10b and *β*-catenin was significantly upregulated in AC010789.1-OE compared with control cells (Figures 5C–F). These data suggest that AC010789.1 may participate in AGA progression by regulating the Wnt/*β*-catenin pathway.

**FIGURE 5:** AC010789.1 targets with Wnt/*β*-catenin signaling pathway to participate in AGA progress. **(A)** The pathway interaction networks with Wnt/*β*-catenin signaling pathway. **(B)** KEGG map of Wnt/*β*-catenin signaling pathway. **(C)** The mRNA expression levels of DKK-1, TGF-*β*1, and Wnt10b in AC010789.1-OE. *n* = 9 **(D–F)** The protein expression levels of TGF-*β*1 and *β*-catenin in AC010789.1-OE. *n* = 3. *p < 0.05, **p < 0.01 and ***p < 0.001.

## Discussion

AGA is an androgen-dependent genetic hair loss disorder characterized by progressive microencapsulation of hair follicles and continuous shortening of the hair follicle growth period (Randall et al., 2000; Rathnayake and Sinclair, 2010). It is currently the most common clinical type of alopecia and can seriously affect a patient’s appearance, mental health, and social behavior. The most common first-line treatments for AGA currently include finasteride and minoxidil, but their application is hindered by limited efficacy, the need for long-term treatment, and inevitable complications. Hair transplant surgery, which involves hair follicle redistribution, is an effective method to improve the appearance of patients; however, as hair follicles cannot be regenerated, AGA patients with large areas of alopecia often have insufficient donor site hair follicles (Rogers, 2015). Therefore, it is necessary to explore the potential molecular mechanisms of AGA onset, progression, and hair follicle regeneration to design more effective treatments.

Several studies indicate that lncRNAs play essential roles in the occurrence and progression of various diseases and that they could be used as new diagnostic and treatment markers. For example, Wang et al. (2018) report that lncHOXA-AS2 promotes the progression of various human tumors by inducing epithelial–mesenchymal transition by directly inhibiting Bax expression, promoting c-Myc and Bcl-2 expression, and activating the Akt-MMP signaling pathway. Accumulating evidence now indicates that the deregulation of the expression of lncRNAs is strongly correlated with the onset and development of AGA (Bao et al., 2017; Zhu et al., 2020). In this study, we used the GSE84839 microarray data set from the GEO database and found that AC010789.1 was expressed to a lower level in AGA scalp tissues than in adjacent normal tissues, which was verified using clinical AGA samples. This suggests that low expression of AC010789.1 is associated with the progression of AGA.

HFSC aging, characterized by a reduction in stemness signatures and a concomitant increase in epidermal commitment, leads to a progressive miniaturization of hair follicles and ultimately, to the hair loss characteristic of AGA (Matsumura et al., 2016). Recently, accumulating evidence indicates that activating HFSCs could be an effective treatment for AGA. Zhang et al. (2020) found that vascular endothelial growth factor significantly reduced 5*α*-dihydrotestosterone-induced HFSC apoptosis by inhibiting the PI3K-Akt pathway, thereby delaying the progression of AGA. Kubo et al. (2020) used fisetin to induce a telogen-to-anagen transition in hair follicles by inducing the proliferation of HFSCs, thus promoting hair growth. Therefore, we hypothesized that AC010789.1 may promote hair growth by promoting the proliferation and differentiation of HFSCs. In the current study, we successfully isolated K15-positive HFSCs from hair follicles of patients with AGA and constructed an AC010789.1-overexpressing HFSC line. K6HF and Lgr5 are shown to be particularly good markers of hair differentiation and proliferation (Roh et al., 2004; Chen et al., 2020b), and we found that the expression of both marker genes as well as the cell proliferation rate were significantly higher in AC010789.1-OE than in the control group, indicating an important role of AC010789.1 in regulating HFSC functions.

Emerging evidence indicates that a large number of lncRNAs participate in a variety of biological functions by interacting with miRNAs and regulating their target genes (Huang, 2018). In this study, we found that AC010789.1 interacts with miR-21 to participate in the progression of AGA. Many reports show that miR-21 plays an essential role in the regulation of several diseases (Lakhter et al., 2018; Wang et al., 2020). To further explore how the interaction between AC010789.1 and hsa-miR-21-5p regulates the pathogenesis of AGA, the GSE36169 microarray data were downloaded, and the genes targeted by hsa-miR-21-5p were identified. A total of 198 AGA-related DEGs, including 11 common genes intersecting with hsa-miR-21-5p target genes, were identified by differential analysis with adjacent normal controls. GO annotation enrichment analysis was performed to explore the biological functions of the AGA-associated DEGs. The upregulated DEGs were primarily enriched in the BP category of immune and inflammatory responses. Previous studies show that an abundance of immune inflammatory cells in the bulge area of the hair follicle leads to the deregulation of the hair follicle microenvironment, thus impairing the normal function of HFSCs and resulting in alopecia (Wang and Higgins, 2020). Interestingly, the downregulated DEGs were directly related to hair follicle development (GO:0001942) and the hair cycle (GO:0042633). Subsequently, we extended the PPI network of the common genes and performed annotated enrichment analysis. Notably, the most downregulated common genes and their most relevant network genes were enriched in angiogenesis. Vascularization is closely related to hair growth (Gentile and Garcovich, 2019). The vascular system plays a vital role in maintaining the HFSC microenvironment, and angiogenesis helps to increase the blood supply of DPCs and promote hair growth. These findings enhance our understanding of the pathogenesis of AGA and the potential mechanism of interaction between AC010789.1 and miR-21-5p to delay the progression of AGA.

The TGF-*β*1 and Wnt signaling pathways are the most crucial pathways for maintaining a quiescent niche and regulating the proliferation and differentiation of HFSCs (Yang and Peng, 2010; Ge et al., 2019). Previous studies report that TGF-*β*1 promotes telogen-to-anagen transition in hair follicles, whereas the transition from anagen to telogen is significantly delayed in the hair follicles of TGF-*β*1 knockout mice (Foitzik et al., 2000; Daszczuk et al., 2020). The Wnt signaling pathway is the main regulatory pathway of biological development and a key driving factor for stem cells in most tissues (Nusse and Clevers, 2017). In the hair follicle, the Wnt signaling pathway plays a key role in starting the hair follicle cycle by initiating the proliferation response of HFSCs in the bulge area; HFSCs treated with Wnt pathway activator can quickly enter the proliferation period (Greco et al., 2009; Hawkshaw et al., 2020). Moreover, Leirós et al. (2017) found that Wnt pathway inhibitors (DKK-1) impair the differentiation of HFSCs, and the addition of promoters (Wnt10b) can reverse this effect in AGA. In addition, miR-21 is closely related to the Wnt/*β*-catenin signaling pathway. Previous studies reveal that inhibiting the expression of miR-21 can lead to upregulation of the Wnt/*β*-catenin pathway, thereby promoting cell activity (Hao et al., 2019; Liu et al., 2019). A recent study also reveals that lncRNA GAS5 competitively combined with miR-21 to regulate the epithelial–mesenchymal transition of human peritoneal mesothelial cells via activation of Wnt/*β*-catenin signaling (Fan et al., 2021). In this study, we conducted a comprehensive pathway analysis of the DEGs, common genes, and the genes most closely related in the PPI network to help us understand the molecular mechanisms underlying AGA progression. In line with our results, we found that the upregulated DEGs were highly enriched in the TGF-*β* signaling pathway, and a majority of the pathways were highly correlated with the Wnt/*β*-catenin signaling pathway. Further analysis showed that AC010789.1 overexpression induced the upregulation of Wnt10b and *β*-catenin, and downregulation of DKK-1 and TGF-*β*1. In summary, our results suggest that AC010789.1 regulates Wnt/*β*-catenin pathway activation, thereby enhancing the proliferation and differentiation of HFSCs and participating in AGA progression.

In summary, our data shows that AC010789.1 overexpression delayed AGA progression through the downregulation of hsa-miR-21-5p and promotion of the Wnt/*β*-catenin signaling pathway (Figure 6). Our findings provide a novel insight into the mechanism by which AC010789.1 promotes the proliferation and differentiation of HFSCs, which sheds light on the future development of lncRNA-based AGA therapies.

**FIGURE 6:** A schematic diagram shows how AC010789.1 delays AGA progression by targeting microRNA-21 and the Wnt/*β*-catenin signaling pathway.

## Data Availability

All datasets generated for this study are included in the article/Supplementary Material, further inquiries can be directed to the corresponding authors.
